# Analysis of College Student Registration Management and Change Prediction Based on Mutated Fuzzy Neural Network Algorithm

**DOI:** 10.1155/2021/7097425

**Published:** 2021-11-16

**Authors:** Yao Wang, Lie Jiao, Chunzhi Liu

**Affiliations:** ^1^Management Science and Engineering, Liaoning Technical University, Fuxin 123000, Liaoning, China; ^2^College of International Business of Shenyang Normal University, Shenyang 110034, Liaoning, China; ^3^Admissions and Employment Guidance Office of Shenyang Normal University, Shenyang 110034, Liaoning, China

## Abstract

Nowadays, a large number of students' academic registrations change every year in universities, but most of these cases are recorded and mathematically and statistically analysed through forms or systems, which are cumbersome and difficult to find some potential information in them. Therefore, timely and effective prediction of student registration changes and early warning of student registration changes by technical means is an important part of university registration management. At present, relevant research is mostly based on mathematical statistical analysis methods such as students' current credit evaluation or course score averages and seldom uses data mining and other technical methods for in-depth research. In this paper, we propose a mutated fuzzy neural network (MFNN) based prediction model for student registration changes in colleges and universities, which can provide supplementary reference decisions for school registration management for school teaching managers. In this paper, we first construct the corresponding prediction model of academic registration variation, define the relevant parameters, and model the optimization problem and propose the objective optimization function. Second, the proposed model is optimized by adding principal component analysis (PCA) to the original model to improve the efficiency of model training and the correct prediction rate. It is verified that the proposed model can effectively predict individual students' academic registration changes with a prediction accuracy of nearly 92.91%.

## 1. Introduction

Currently, the popularization of education has been deeply popularized, and the proportion of enrolment in colleges and universities is increasing year by year, so the traditional offline manual student management has long been unable to meet today's needs, and online student management systems have been born and commonly used [1–4]. However, in the face of the increasing number of students, the academic affairs center, as the core department of school teaching management, faces increasingly severe management challenges, especially in the management of student registration, which is an important identification of students in school, marking a student's affiliation with a school and a major, and recording the whole process of a student from the beginning to the end of the school year [5].

Good academic registration management is of far-reaching significance to the overall teaching management of colleges and universities, and it is inseparable from students' study, graduation, and future work [6–8]. According to the research, every year, a large number of students' academic registrations are changed in every university, and in response to this phenomenon, the way of “dealing with academic registrations after they are changed” is no longer used, and most universities have established a certain early warning system for academic registrations, that is, in the management of students' academic registrations, students are informed of their bad behaviours in their studies in time. The mechanism is mostly based on systematic data recording and mathematical statistical analysis of students' failing scores in examinations and the number of failed courses to achieve the prediction of early warning effect. To a certain extent, this approach is cumbersome and difficult to detect certain potential information and patterns in it, and it can only analyse the student's academic status variation from a small latitude [9]. For students, some of them cannot even grasp by themselves whether they can finish their studies normally or not, so it is an important task of teaching management in universities to make multidimensional and effective prediction of student's academic registration changes by using technical means [10–12].

There are still many problems in the construction of the early warning mechanism of university status. In the current management mechanism, student status changes are mainly determined by the student's course grades and passing status. This kind of examination result is regarded as the only judgment method, which makes it easy for students to speculate for examinations and do not pay attention to the development of their own comprehensive qualities. In most cases, the early warning is given only after the students have failed multiple exams. From the perspective of time, it is not possible to take timely assistance and remedial measures to the students, and the effect of taking precautions cannot be achieved. At the same time, as the enrolment scale of colleges and universities is gradually expanding, the provision of academic administration management personnel may not be able to keep up with the growth rate of the number of students in a timely manner. As a result, academic administration administrators are often not in the daily management of university academic affairs and have no time to take into account the existing status of student status changes. It is often just a formality, but it is impossible to think and discuss deeply. It is only a means to give the students the treatment results according to the form, but it is not the essence of management. It is necessary to implement planned assistance work for the students being treated. Only continuous supervision can really help students find and solve problems in school.

In order to achieve the research objectives, this paper is divided into the following five sections: Section 1 conducts a background research on the current university academic affairs management, especially the academic registration variation management, and conducts an in-depth investigation on the shortcomings in the academic registration variation management affairs, and clarifies the practical significance of this research.  Section 2 investigates the current research status of academic registration variation and the research status of the adopted neural network algorithm and clarifies the main research directions and innovation points of this paper.  Section 3 proposes to build a prediction model based on MFNN algorithm and optimize the prediction model by using PCA to achieve more accurate prediction and practical application of student registration variation in colleges and universities and introduces the adopted cross-validation method and then validates and evaluates the prediction effect of the MFNN algorithm-based student registration variation model and the optimized model, respectively. The analysis of the prediction results illustrates its usefulness in assisting teaching management decisions.  Section 4 summarizes the work of this paper and clarifies the practical significance of the MFNN algorithm-based student registration variation model in the application of student registration variation prediction in colleges and universities and reflects that there are still aspects that need to be further researched to provide a reference direction for future research work on student registration variation management in colleges and universities.

## 2. Related Work

Academic registration is a decree status of a student belonging to a particular school [13]. Some countries with early start and rapid development of higher education have been developing and innovating university management [14]. Since the end of the eighteenth century, the credit system has been proposed by some universities and gradually recognized by the educational circles of various countries, and its development to today, the credit system in school registration management has been transformed into a full credit system, that is, students can graduate after completing a certain number of credits, and if there is a course failure, the credits of the course will be zero, and students have certain authority to choose to retake the course or choose. For each course taken, students need to pay tuition for one course, i.e., tuition is charged according to the credits taken. This has somewhat weakened the concept of early warning of academic registration changes, which generally does not occur unless there are other external reasons such as personal or family reasons. With the change of education status, the number of students enrolled in colleges and universities increases gradually every year, and the content and way of teaching management in colleges and universities have changed, from the traditional offline manual management records to the development and operation of online information management system, which has solved the problem of expanding the content and simplifying the related process of academic affairs management to a certain extent, and has initially adapted to the current status of college education. In the face of the phenomenon that the number of students' academic registration changes gradually increases in each university every year, each university has considered and put forward the corresponding early warning mechanism of academic registration changes accordingly. Scholars such as Smolyakova et al. mentioned in related literatures that several types of early warning mechanisms should be constructed for students' changes in their school status throughout their learning career in order to achieve a comprehensive early warning effect for their learning stage [15]. For example, school opening warning, grade warning, withdrawal warning, and graduation warning that are also adopted by most colleges and universities for academic variation warning management [16]. Warren et al. have proposed to analyse the teacher evaluation data, find out the academic style problems of each class, discover potential academic early warning objects, and establish a new academic variation early warning mechanism [17]. Wei et al. proposed to use association rule technology to build a student grade warning model only for student grades. The early warning model of students' grades can be used to determine whether students have the possibility of repeating or withdrawing from school through early warning of grades [18]. Xiang et al. have analysed the important role of data mining methods in the early warning system of college student status management, and data mining methods can be used to discover unknown or potential rules in the educational administration center database [19]. Xiang has proposed the idea of constructing a corresponding teaching early warning system based on Internet + [20]. In addition, Xin has studied the construction of corresponding teaching early warning systems based on Internet + [21]. Yang adopted an open attitude and dynamically mine the hidden indicators behind the students' evaluation of teachers' teaching data [22].

Most of the relevant early warning mechanisms in universities are based on mathematical and statistical analysis such as students' current credit ratings or course grade averages, and there is basically no extensive and in-depth research on the management of student's academic status changes using technical methods such as data mining [23–25].

In order to better manage the status of college students and predict the changes, this paper attempts to conduct a study on the prediction of college students' academic registration variation. By using the data of students of a university from 2014 to 2018 class, we extracted the dataset of student academic registration variation research after analysing the data in a multidimensional way, and proposed to build a prediction model of academic registration variation based on neural network algorithm by comparing the algorithms used for prediction applications. Based on this, the model is evaluated in terms of its effectiveness in predicting student registration variations using a multi-round cross-validation method. After the evaluation, the model can better predict the student's academic registration changes in universities. Meanwhile, considering the improvement of the accuracy of the model in predicting student registration changes, the optimization of the model was completed by using principal component analysis and sensitivity analysis methods, which in turn improved the prediction effectiveness of the model.

### 2.1. Prediction Model of School Registration Variation Based on MFNN Algorithm

Most of the current researches on academic registration variation in colleges and universities stay in establishing a certain academic registration early warning mechanism, which mostly analyses students' daily performance and examination results statistically and uses manual system entry for monitoring and early warning, which is complicated to operate and has to invest more manpower [26]. This section combines the above research status, proposes a prediction model of school registration variation based on MFNN, based on the characteristics of the MFNN algorithm, and reasonably trains the neural network to achieve the effect of effectively predicting student registration variation, providing managers with auxiliary decision-making and reducing manual pressure.

### 2.2. Construction of a Prediction Model of School Registration Variation Based on the Combination of MFNN and T-S Fuzzy Model

Neural network thinking assumes that the animal brain is a complex learning system for recognition through the tight interconnection of neurons [27–32]. Although the structure of individual neurons is relatively simple, the dense network formed by connecting these neurons can perform complex learning tasks such as pattern recognition and classification. Considering the influence of nonlinear combinatorial modeling ability and generalization ability on prediction results in certain environments, the MFNN algorithm is chosen in this paper to study and predict the student's academic registration variation in colleges and universities.  Figure 1 shows a fuzzy neural network model constructed with a T-S architecture, where the back network is used to generate fuzzy rules while the front network is used to match the generated fuzzy rules with each layer.

First, the posterior network for generating fuzzy rules is a network layer divided according to the specific problem, and these network layers are juxtaposed with each other, with each subnetwork layer eventually producing a desired output quantity, starting with a single output network as an example. The first layer is the input layer, which feeds the input variables into the neural network system, corresponding to the hydraulic fluid pressure setting or the pressure injection speed setting and the feedback deviation corresponding to the setting value in this paper. The second layer has *L* nodes, one for each fuzzy rule, and the function of this layer is to calculate the rules needed for the next iteration of the neural network, i.e.,

(1) $$\begin{array}{c} y_{j}=c_{0}j+c_{1}j_{1}+\cdots +c_{n}^{j}x_{j}=\sum_{i=0}^{L}c_{i}^{j}x_{j}\;\left(j=1,\ldots ,L\right), \end{array}$$

where *n* is the dimension of the input variable, *j* is the number of nodes in the second layer, and *y*_*j*_ is the output of the fuzzy rule in the second layer. The third layer is the final desired output, i.e.,

(2) $$\begin{array}{c} y=\sum_{j=1}^{L}f_{j}y_{j}, \end{array}$$

where *f*_*j*_ is the fitness weight of each fuzzy rule and the output of the third layer. The final output is the sum of the posterior and anterior rules after weighting, and the output of the anterior network corrects the connection weights of the final third layer of the posterior network.

As a correction to the front network of connection weights, unlike the back network, the number of layers of the front network is fixed, consisting of four layers, the first layer of the front network is also the input layer to pass the input variables to the next layer, for this system the number of nodes in this layer is 2, each node in the second layer corresponds to a fuzzy control language variables, which is the fuzzy language description required by the system, here the fuzzy language description is chosen as follows:

  E is the domain of the argument for [−1,1]
  E is the fuzzy rules of {NB, NM, NS, ZO, PS, PM, PB}
  EC is the domain of the argument for [−1,1]
  EC is the fuzzy rule of {NB, NM, NS, ZO, PS, PM, PB}

The role of this layer is to calculate the affiliation function *μ*_*i*_^*j*^ (Gaussian affiliation function), which determines all degrees of each fuzzy variable to the input variables, where

(3) $$\begin{array}{c} \mu_{i}^{j=e}e^{-\left(x-c\right)2/\sigma }, \end{array}$$

where 1,2,…, *n*, *j*=1,2,…, *m*_*i*_, *m*_*i*_ is the number of fuzzy partitions of *x*_*i*_, *μ*_*i*_^*i*^ is a Gaussian affiliation function, and the number of nodes in the second layer is ∑_*i*=1_^*n*^*m*_*i*_.

Each node in the third layer of the network corresponds to a fuzzy rule, and the fuzzy rule is evaluated for each iteration, both calculating the fitness function of each rule, which can be expressed as *α*_*j*_=*μ*_*i*_^*i*1^*μ*_2_^*i*2^ … *μ*_*m*_^*im*^, and the total number of nodes in this layer can be seen as *m*. For a system with a certain input value, the affiliation function of fuzzy linguistic variables far from the input point will be small while for the affiliation function will become larger and larger as the distance gets closer to the fourth layer serves to normalize the calculation of the connection weights, i.e.,

(4) $$\begin{array}{c} \bar{\alpha_{j}}=\frac{\alpha_{j}}{\sum_{j=1}^{m}\alpha_{j}}, \end{array}$$

where *a*_j_ is the adaptation function corresponding to the first *j* rule.

### 2.3. Optimization Problem Modeling

In any experimental study, one takes certain measures in order to measure, under certain constraints, whether the parameters that are the focus of the study being done have reached their optimal values using one criterion, which leads to the optimization problem. Optimization refers to finding the optimal solution for a quantifiable optimization problem by finding the optimal solution within a reasonable time frame. This process is crucial in the research process. The first step in solving an optimization problem is to construct a mathematical model to describe the optimization problem to be addressed, which in general is as follows.

Given a function *g* : *P*⊆*R*^*m*^⟶*R*, *P* ≠ ∅, when and only when *x*^*∗*^ ∈ *P*, ∀*x* ∈ *P* : *g*(*x*^*∗*^) ≤ *g*(*x*), then the function value *g*^*∗*^ : =*g*(*x*^*∗*^) > −*∞* is the minimum, where *g* is the objective function and P is the set of feasible regions. From this, it is clear that every optimization problem contains the following basic elements:

(1) The objective function, which indicates the quantity to be optimized, in this study is the accuracy of predicting the student's academic registration variation in the sample set, and the formula is
  (5) $$\begin{array}{c} \text{accuracy}=\frac{{\text{num}}_{\text{corret}}}{N}, \end{array}$$
where num_correct_ is the number of students whose academic records are correctly predicted and N is the total number of data samples in the training set.
(2) Unknown parameters or variables, indicating that these parameters or variables will have an impact on the objective function, which in this study are mainly the number of input units, the number of hidden units, and the back-propagation error calculation method. In the later sections, the focus on optimization of these variables is mainly completed.
(3) Constraints, indicating the conditions used to constrain the values of unknown parameters or variables.

Therefore, it is an important direction in the research field that has both theoretical significance and practical application value to focus on optimization problems in practice and use related technologies to improve the algorithm and continuously expand the practical application scope of the algorithm and improve the algorithm system.

### 2.4. PCA-Optimized Prediction Model for Academic Variance

When performing data mining tasks, the database used will contain a large number of records and variables associated with the records, but not all of these variables are independent and uncorrelated with each other. Predictor variables that are strongly correlated will cause instability in the network training, which will lead to unstable results. Moreover, if too many initial predictor variables are defined, the network model will become complicated and difficult to solve during the training process, which in a way violates the principle of parsimony, so it is necessary to limit the number of predictor variables.

The dataset of this study was obtained from the academic affairs management system of a university, in which there were 13 database tables related to students, as detailed in Table 1.

In this study, the number of input units, i.e., the number of predictor variables, is set to 16 for the MFNN model, which can be considered to compress the number of variables so that the information contained in the 16 variables can be basically included even if fewer variables are used. Therefore, it is proposed to reduce the dimensionality of the predictor variables by using PCA. By transforming the original 16-dimensional space, N (*N* < 16) mutual orthogonal bases are found sequentially to approximate the original 16-dimensional space, so that the training dataset has a large variance on all these N orthogonal bases, thus realizing the dimensionality reduction of the original space and minimizing the loss of information data.

There are 2000 training data *x*_1_, *x*_2_,…, *x*_2000_ containing 16 predictor variables in the study dataset, the training data matrix is *X*=[*x*_1_, *x*_2_,…, *x*_2000_] , the final projection vector is *e*, and the original data center point is

(6) $$\begin{array}{c} w=\frac{1}{2000}\sum_{i=1}^{20000}x_{i}. \end{array}$$

The variance of the training data after projection is

(7) $$\begin{array}{c} D=\frac{1}{2000}\sum_{i=1}^{2000}{\left(e^{T}x_{i}-e^{T}w\right)}^{2}, \end{array}$$

(8) $$\begin{array}{c} \begin{array}{c} D=e^{T}\left(\frac{1}{2000}\overset{2000}{\underset{i=1}{\sum }}\left(x_{i}-w\right){\left(x_{i}-w\right)}^{r}\right)w \end{array}. \end{array}$$

Calculating the covariance matrix *M*=1/2000∑_*i*=1_^2010^(*x*_*i*_ − *w*)(*x*_*i*_ − *w*)^*T*^, equation (8) is converted to

(9) $$\begin{array}{c} D=e^{T}Me. \end{array}$$

To find the optimal projection vector is to calculate **D** the maximum value, and the extreme value can be obtained by using the Lagrange multiplier method:

(10) $$\begin{array}{c} Me_{i}=\lambda_{i}e_{i},\;i=1,2,\ldots ,16. \end{array}$$

From (10), the eigenvector of the covariance matrix *M* is *e*_*i*_. So the steps to reduce the dimensionality of the original dataset using PCA are as follows:

1. Calculate for the dataset and obtain the covariance matrix *M*
2. Obtain the eigenvalues, and the corresponding eigenvectors, by decomposing the covariance matrix *M*
3. Sort the eigenvalues from the largest to the smallest
4. The first *t* eigenvector is the desired *e*_1_, *e*_2_,…, *e*_*t*°_
5. Then the first principal component is a linear combination *Y*_1_=*e*_1_*X*, and so on

The selection of the number of predictor variables in the final training dataset after dimensionality reduction is also an important factor affecting PCA dimensionality reduction. Usually, the components are selected in order of their variance contribution ratio, and the calculation formula is

(11) $$\begin{array}{c} \text{ratio}=\frac{\sum_{i=1}^{k}\lambda_{i}}{\sum_{i=1}^{16}\lambda_{j}}. \end{array}$$

Following the above steps, the 16 predictor variables in the dataset of the Academic Variance Study were analysed, and the partial component matrix is shown in Figure 2. Each column in Figure 2 represents one of the components F, and the elements in the column are the correlation weights of each component, i.e., the correlation coefficients of the covariates.

Usually the first principal component can be used as the best summary of the predictive correlation of academic variance, and from the partial component figure above, it can be seen that the average grade in planned courses/public courses, planned courses, average grade in elective courses, and average assessment grade in English extension courses all have relatively similar component weights, and this predictor variable is highly correlated with the first principal component compared to the other components. By calculating the proportion of variance contribution and cumulative contribution of each component, the results are presented in Figure 3.

As can be seen in Figure 3, the first and second principal components contribute 30% and 25%, respectively, which is equivalent to containing half of the information of the original 16 predictor variables. And the last two components basically do not contribute any valid information. Therefore, for the extraction of the number of principal components, we can refer to the general experience and select the *n* principal components with a cumulative contribution ratio >85% as the total number of features in the final training dataset, i.e., the first seven principal components are selected as the research dataset after dimensionality reduction in this study. For this network prediction model, the number of input units is defined as 7, and the number of output units is defined as 3. The dimensionality of the study dataset after dimensionality reduction is greatly compressed compared with the previous study dataset, which can greatly improve the training speed of the neural network model.

## 3. Model Prediction Validation and Example Application

This section will use the K-fold cross-validation method to verify the prediction effects of the above-mentioned construction models. First, the K-fold cross-validation method will be introduced, and then the prediction results of the initially constructed student status change prediction model based on the BP neural network algorithm will be verified and analysed. The optimized prediction model for student status changes is verified. Finally, the optimized prediction model for student status changes is applied to the prediction of student status changes in colleges and universities. The analysis results show the effectiveness of the model in actual college student status management.

### 3.1. K-Fold Cross-Validation Method

In order to realize the evaluation of the validity of the MFNN-based prediction model for student status changes proposed in this paper, the K-Fold Cross-Validation Method (KFCVM) is used in this paper. KFCVMC is a technique used to evaluate the effect of a learning model on an independent dataset, and is usually used to assess the accuracy of the model prediction and the actual effect of the application. The results of the test set are averaged as the final actual results through *K* times of cross-training and testing. The specific process description is summarized as follows:

1. The *T* training set is divided equally into *k* disjoint subsets, and the number of training samples in *n* each subset is *n*/*k* assumed *T* to be, and the corresponding subset is called {*t*_1_, *t*_2_,…, *t*_*k*_}
2. From the split set, extract one at a time as the test set and the rest as the training set
3. Apply the test set to the model trained by the training set to obtain the correct classification results
4. Calculate the average result of the correct classification rate obtained for each time and treat it as the true correct classification of the model *k*

The calculation formula is

(12) $$\begin{array}{c} \text{accuracy}=\frac{1}{k}\sum_{i=1}^{k}\frac{{\text{Corr}}_{i}}{n_{\text{tet}}}, \end{array}$$

where Corr_*i*_ denotes the number of samples finally classified correctly in the first *i* test set *n*_test_ and is the total number of samples in the test set. The general trifold cross-validation schematic is shown in Figure 4.

In this study, *K* = 5, i.e., the number of data in the training set is 1600 and the number of data in the test set is 400, and five rounds of cross-validation are conducted. In each round of validation, the number of iterations of the network model is set to 1000, and the training set is used to train the model repeatedly until the maximum number of iterations is reached, and then the test set sample data are fed into the trained network prediction model one by one to obtain the prediction results, and the results are compared with the actual classification results of the test set data. The overall correct prediction rate in the validation round is obtained. Therefore, based on the above definition, the final average correct rate of the prediction of student's school registration variation by combining the nondeterministic parameters when the number of hidden layers based on the MFNN model is 6, 7 and 8 is shown in Figures 5–7, respectively.

From Figures 5–7, it can be seen that when the number of hidden layers is 7, the overall correct rate of student registration prediction is high, basically above 80%. Among them, when the learning rate is 0.05 and the momentum term is 0.3, the correct prediction rate for student registration variation is the highest, reaching 84.75%, which basically proves the feasibility of applying the MFNN algorithm-based student registration variation prediction model to student registration variation prediction.

Then, the initial research dataset was downscaled using PCA, and after the downscaling process, the first 7 principal component data were selected to replace the initial research dataset as the new input variables for the training and prediction of the network model. Based on the existing optimization, the variance contribution ratio and the cumulative contribution ratio of each component can be obtained by dimensionality reduction of 13 variables using PCA again on this basis, and the specific results are shown in Figure 8.

The number of output units of the network prediction model based on mutation fuzzy neural network algorithm is redefined as 7, the number of output nodes is still 3, the number of hidden layer units is 3–5, and the learning rate and momentum terms are 0.08 and 0.25, respectively. The remaining settings remain unchanged.  Figure 9 shows the final average accuracy of the network model before and after the combination of values predicting student registration changes.

From Figure 9, it can be seen that when the number of hidden layers is 5, the optimized network model has the highest correction rate of predicting a pair of student's academic registration changes, which can reach 92.91%, and the average correct rate of prediction is improved by about 4% compared with the previous network prediction model without optimization.

## 4. Summary and Outlook

Based on the current situation of student registration variation management in universities, this paper proposes to design an MFNN algorithm-based student registration variation prediction model to predict and realize the auxiliary management of student registration. It has been verified that the model can effectively predict the changes of individual students' school status, and the prediction accuracy rate is close to 92.91%. It is proved that the model is effective in predicting the student registration variation and can assist the academic administration workers to make some decisions in the management of student registration variation to a certain extent. The present research work on academic registration variation management in colleges and universities only implements a student registration variation prediction model from the technical perspective and optimizes the model to prove the effectiveness of the prediction model applied to student registration variation prediction, but it is far from enough and there is still much room for research.

## Figures and Tables

**Figure 1:** The T-S model combined with neural network architecture.

**Figure 2:** The partial component matrix.

**Figure 3:** The proportion of variance contribution and cumulative contribution of each component.

**Figure 4:** The trifold cross-validation diagram.

**Figure 5:** The prediction results of nondeterministic parameter combinations when the number of hidden layers is 6.

**Figure 6:** The prediction results of nondeterministic parameter combinations when the number of hidden layers is 7.

**Figure 7:** The prediction results of nondeterministic parameter combinations when the number of hidden layers is 8.

**Figure 8:** The proportion of variance contribution and cumulative contribution of each component after PCA optimization.

**Figure 9:** The comparison of prediction results before and after PCA optimization.

**Table 1:** The database tables related to student data.

Table Name	Fields
course__category	Category ID, category name
department	Faculty code, faculty name
major	Major code, major name
filed	Direction code, direction name
coursejibraty	Course ID, course number, course Chinese name, credits, total hours, lab hours, course scope, for grade, for department
course	Course semester, course class number, course ID
school_class	ID, type, number, name
student	Student number, name, gender, current credits, student type, faculty, major, direction, grade, class
student__category	ID, type name
student__score	ID, student number, course ID, serial number, semester year, course class ID, regular grade, grade, course category, nature of exam, grading system
change__category	Code, name
change_type	Code, name, nature, type of student
student__change	ID, student number, nature of academic registration change, type of academic registration change, semester of academic registration change, date of academic registration change

## Data Availability

The data used to support the findings of this study are available from the corresponding author upon request.
